# Overweight and Obesity and their Association with Dietary Habits, and Sociodemographic Characteristics Among Male Primary School Children in Al-Hassa, Kingdom of Saudi Arabia

**DOI:** 10.4103/0970-0218.42058

**Published:** 2008-07

**Authors:** Tarek Tawfik Amin, Ali Ibrahim Al-Sultan, Ayub Ali

**Affiliations:** Department of Family and Community Medicine, College of Medicine, King Faisal University-Al Hassa, Saudi Arabia; 1 Department of Internal Medicine, College of Medicine, King Faisal University-Al Hassa, Saudi Arabia

**Keywords:** Body mass index, childhood obesity, dietary habits, Saudi Arabia

## Abstract

**Objectives:**

To assess the magnitude of obesity and overweight among male primary school children, and to find the possible association between obesity/overweight and dietary habits and sociodemographic differentials among them.

**Study design and Methods:**

A cross-sectional descriptive study, including 1139 Saudi male children enrolled in the 5^th^ and 6^th^ grades in public primary schools in Al Hassa, Kingdom of Saudi Arabia (KSA), was conducted. The test included a multistage random sampling technique, based on interview using Youth and Adolescent Food Frequency Questionnaire, gathering data regarding dietary intake, dietary habits, followed by anthropometric measurements with the calculation of body mass index (BMI), the interpretation of which was based on Cole's tables for the standard definition of overweight and obesity. Sociodemographic data were collected through a parental questionnaire from. Data analysis was performed using the SPSS 12 software (SPSS Inc. Chicago, IL, USA); both univariate and multivariate analyses were performed.

**Results:**

The age of the school children ranged from 10–14 years. The prevalence of overweight among the subjects was 14.2%, while that of obesity was 9.7%; the prevalence was more in the urban, older age students. The mothers of obese and overweight children were less educated and more working. Missing and or infrequent intake of breakfast at home, frequent consumption of fast foods, low servings per day of fruits, vegetables, milk and dairy products, with frequent consumption of sweets/candy and carbonated drinks were all predictors of obesity and overweight among the schoolchildren studied.

**Conclusion:**

The prevalence of childhood obesity is escalating and approaching figures that have been reported till now from the developed countries. Less healthy dietary habits and poor selection of food may be responsible for this high prevalence.

## Introduction

Obesity is becoming a worldwide problem affecting all levels of society and is thus being described as a global epidemic.(1) On one hand, the highest rates of childhood obesity have been observed in the developed countries, its prevalence is increasing in the developing countries also. The prevalence of childhood obesity is high in the Middle Eastern, Central and Eastern European countries.(2) For example, Iran has been reported to be one of the seven countries with the highest prevalence of childhood obesity;(3) in Saudi Arabia, one in every six children aged 6–18 years old is obese.(4)

The numerous psychological, physical and economic consequences of obesity are well known. Childhood obesity affects self esteem and has negative consequences on the cognitive and social development.(5,6) Conditions such as type 2 diabetes mellitus, hypertension, and hypercholesterolemia, which were noted primarily in adults, are becoming more common among children with the increase in the prevalence of obesity.(7) Because childhood obesity often persists until adulthood, an increasing number of adults will be at an increased risk of these conditions as well as of cardiovascular disease, osteoarthritis and certain types of cancer.(8,9)

Overall, the obesity epidemic results in a substantial decrease in the quality of life and life expectancy, and it accounts for heavy expenditure in provision of health care.(10) Due to difficulty in the treatment of obesity in adults and the many long-term adverse effects of childhood obesity, prevention of childhood obesity has now been recognized as a public health priority.(11)

In many developing countries, the progression of nutritional transition has been detected, characterized by a reduction in the prevalence of nutritional deficiencies and the more expressive occurrence of overweight and obesity not only in the adult population but also among children and adolescents;(12) these characteristics are fundamentally associated with changes in lifestyle and eating habits.(10)

Food intake has been associated with obesity not only in terms of the volume of food ingested but also in terms of the composition and quality of diet. Furthermore, eating habits have also changed and current habits include low consumption of fruits, green vegetables, and milk; increasing consumption of snacks, sweets, and soft drinks; and skipping breakfast; these eating habits result in continuous increase in adiposity among children.(12) Eating habits in addition to environmental differentials represent the most dominant determinant in increasing the tendency of overweight and obesity among children,(13) and a modification in the eating habits may be singleton tactic strategy to a more appropriate weight control.(14)

Several studies were carried out to assess the prevalence of overweight and obesity among Saudi Arabian children;(4,15–16) however, very few have assessed the association between eating habits, sociodemographic differentials and obesity in these children(17) compared to those obtained from the developed countries. This study provides the baseline information for future comparison regarding the possible factors underlying the high prevalence of childhood obesity among primary school children in Al-Hassa, Kingdom of Saudi Arabia (KSA). In addition, such information may be of value in developing programs and policies to combat the epidemic of childhood obesity among primary school children in KSA.

The objectives of this study were to assess the magnitude of obesity and overweight among male primary school children, and to find a possible association between obesity/overweight and dietary habits and the sociodemographic differentials among them.

## Population and Methods

### Setting

The study was carried out in Al-Hassa Governorate located in the Eastern province of Saudi Arabia. The total number of public primary schools was 160; of these, 25 were Hegar ‘Bedouin scattered communities’; 88, urban and 47, rural.

According to the local Directorate of Education, the total population of children enrolled in these schools was 44408. We selected students from the 5^th^ and 6^th^ grades for a better communication. The recorded total number of students enrolled in these grades was 12432. Hegar schools were excluded for convenience in the transportation process. The schools in the urban areas were located in two districts, namely, ‘Hofuf’ and ‘Mubraz’, and each district is divided into five localities. Schools in the rural areas were located in the Northern and Eastern villages; we identified six major villages.

### Study design and sampling

A cross-sectional study was conducted, assuming the expected frequency of obesity among this age group as 16%(4) and the worst acceptable frequency as 15%, from the total population in this age group (12432) with a 95% confidence and 80% power; the total estimated sample size should include 1065 subjects.

To overcome the sampling error by using cluster sampling technique, 20% more participants were included, and the total final sample size comprised 1278 males. A proportionate stratified sampling method was applied with regard to the rural/urban distribution.

An updated list of all public primary schools was used as the sampling frame. The schools were stratified proportionately according to urban/rural distribution; 16 schools were randomly selected of which 6 were rural and 10 were urban schools.

According to Saudi community traditions, male investigators are not permitted to access female students; in addition, no female investigators were recruited during the conduction of this study at our institution.

#### Data collection tools and techniques:

After a brief orientation, selected school children were subjected to the following experiments:

#### 1- Anthropometric measurements:

The weight was measured using a commercial scale (Seca, Germany) with an accuracy of ±100 g. The subjects asked to remove their footwear and wear minimal clothes before weighing them. The standing body height was measured to the nearest 0.5 cm by using a commercial stadiometer with the shoulder in a relaxed position and arms hanging freely and without shoes. The scales were recalibrated after each measurement. All measurements were carried out outside the class room on individual and solicited bases after an interview with food frequency questionnaire.

Body mass index was (BMI) calculated as ‘body weight in kilograms/height in meters’;(2) we applied the cut-off points recommended by Cole *et al*,(18) in identifying the age and gender-specific cut-off points for the BMI with the age ranging from 1 to 18 years for the diagnosis of overweight and obesity among the included subjects.

Children with ≥85 percentiles were considered overweight, those with ≥95 percentiles were obese, while those with <85 percentiles were considered desirable or lean.

#### 2- Sociodemographic and dietary data:

Two forms were used for gathering data regarding

(1) Food intake and dietary habits were assessed through a personal interview using items from the validated Youth and Adolescence Food Frequency Questionnaire.(19,20) This diet assessment instrument was developed in a multiethnic sample of US children. The alpha coefficient for nutrients ranged from 0.26 for protein to 0.57 for calcium; for food, this coefficient ranged from 0.39 for meat to 0.57 for carbonated soft drinks. Food intake was assessed as servings per day by multiplying the average portion size by the frequency of intake. Inquiries regarding food habits using closed-ended questions were added, which included the following: taking breakfast at home, frequency of breakfast in the last week, consuming food at school and the frequency of consumption of fast foods one week before the interview. The students were interviewed by two well-trained assistants under the supervision of the investigators.

The field pretest was conducted for testing the contents, phrasing and sequencing of the procedure by enrolling 150 primary school children other than those in the sample from nearby primary schools.

(2) Sociodemographic data were collected using a parental form and included the following items: current residence, date of birth, parental educational and occupational status and family size. These formats were sent to the guardians at home to complete.

#### Data management and data processing:

The original total population sampled was 1282, but for data validity, 143 subjects were excluded due to low responses from parents in submitting the completed sociodemographic data. The students excluded from the analysis did not significantly differ form those included with regard to the distribution of BMI or dietary habits.

Data entry and data processing were carried out using the SPSS version 12 software (SPSS Inc. Chicago, Illinois, USA). Both the descriptive and inferential data analyses were applied using the appropriate statistical tests of significance (chi-square, *t*-test). A multivariate binary logistic regression model was generated by including significant variables in the univariate analysis. Two models were created; the first dealt with the sociodemographic and dietary habits, while the second was used to define the possible food items for the prediction of obesity and overweight.

Confidence interval of 95% and significant difference of ≤0.05 was found to be valid and convenient.

#### Ethical considerations:

Permission was obtained from the authorities of the local School Health and Education Directorate. The teaching and administrative school staff underwent prior orientation. Before commencing the procedures of interviewing and measurements, the students underwent a brief orientation.

## Results

A total of 1139 male primary school children were included with their age ranging from 10 to 14 year (mean age, 11.91 ± 1.00 years); 62.1% of the students included resided in urban areas.

Prevalence of obesity and overweight: Of the 1139 male schoolchildren from a Saudi primary school, 110 (9.7%, 95% confidence intervals, CI = 8.1–11.5%) were obese with regard to age-/gender-specific BMI, and 162 (14.2%) were overweight (CI= 12.3%–16.4%).

The number of overweight and obese children was higher in urban schools, among the older age group (Odds ratio, OR = 2.2), belonged to less educated parents, more working mothers and small family size (*P* = 0.001) as compared to their counterparts with a desirable BMI [Table 1].

**Table 1:** Sociodemographic and anthropometric sample characteristics in relation to the BMI classification

Anthropometry and sociodemographic variables	Body mass index classification		Univariate analysis odds ratio (95% CI)* and *P* value
		
	Total (N = 1139) No. (%)	Overweight and obese children (N = 272) No. (%)	
Weight in kg (mean ± SD)	42.4 ± 6.7	56.6 ± 11.7	*P* = 0.001*†
Height in cm (mean ± SD)	148.8 ± 7.5	151.6 ± 8.7	*P* = 0.001*†
Age in years (mean ± SD)	11.8 ± 0.8	12.1 ± 0.9	*P* = 0.001*†
Body mass index (mean ± SD)	20.8 ± 6.4	27.7 ± 6.9	*P* = 0.001*†
<85th percentiles	867 (76.1)	-	1.6 (1.2–2.1)*
≥85th to <95th percentiles	-	162 (14.2)	1 (ref)
≥95th percentiles	-	110 (9.7)	0.7 (0.5–0.9)*
Residence:			
Urban	707 (62.1)	190 (26.9)	1 (ref)
Rural	432 (37.9)	82 (19.0)	0.5 (0.4–0.7)**
School grade:			
5^th^ grade	442 (38.8)	90 (20.4)	2.2 (1.7–3.1)**
6^th^ grade	697 (61.2)	182 (26.1)	1 (ref)
Age groups:			
10–12 years	419 (36.8)	72 (17.2)	1.5 (1.1–2.1)*
12–14 years	665 (58.4)	197 (29.6)	1.3 (0.9–1.7)
14 years	55 (4.8)	3 (5.5)	0.9 (0.6–1.2)
Mother's education:			
Illiterate/read and write	234 (20.5)	70 (30.0)	1 (ref)
Primary/preparatory	415 (36.4)	111 (26.7)	1.9 (1.2–2.9)*
Secondary	232 (20.4)	50 (21.6)	0.6 (0.5–0.9)*
University/higher	258 (22.7)	41 (15.9)	1.0 (0.7–1.3)
Father's education:			
Illiterate/read and write	111 (9.7)	39 (35.1)	1 (ref)
Primary/preparatory	392 (34.4)	73 (18.6)	1.7 (1.2–2.4)**
Secondary	295 (25.9)	69 (23.4)	1 (ref)
University/higher	341 (30.0)	91 (26.7)	1.9 (1.2–3.2)*
Working Mother:			
Yes	209 (18.3)	67 (32.1)	0.3 (0.2–0.4)**
No	930 (81.7)	205 (22.0)	1 (ref)
Working Father:			
Yes	1006 (88.3)	252 (25.0)	-
No	133 (11.7)	20 (15.0)	-
Family size:			
>6 per family	709 (62.2)	109 (15.4)	-
≤6 per family	430 (37.8)	163 (38.0)	-

* *P* < 0.05

† =*t*-test

** *P* < 0.01. (95% CI) = 95% Confidence Interval, (ref) = reference group

Dietary habits of the included students: The frequency of eating breakfast at home in the last week, before and on the day of the interview was significantly high among lean children compared to overweight and obese peers.

The frequency of eating out was high among overweight and obese children with an OR increased from 0.2 for low frequency to >4 for a frequency of 5 times per week or more (*P* < 0.001) [Table 2].

**Table 2:** Some dietary habits as stated by the included primary school children associated with their BMI classification

Dietary habits	Body mass index classification		Univariate analysis odds ratio (95% CI)* and *P* value (N = 867) No. (%)
		
	Obese and overweight	Nonobese/nonoverweight (N = 272) No. (%)	
Dietary habits:			
Breakfast at home (frequency/last week):			
Daily	75 (27.6)	441 (50.9)	1 (ref)
3–6 times/week	87 (32.0)	134 (15.4)	2.6 (1.9–3.6)**
<2 times/week	110 (40.4)	258 (29.7)	1.6 (1.2–2.2)**
Taking breakfast at home on the day of interview:			
Yes	142 (52.2)	753 (86.9)	1 (ref)
No	130 (47.8)	114 (13.1)	6.1 (4.4–8.3)**
Eating at school (frequency/last week):			
Daily	175 (64.3)	502 (57.9)	1 (ref)
3–4 times/week	16 (5.9)	107 (12.3)	0.4 (0.3–0.8)*
<2 times/week	81 (29.8)	258 (29.8)	1.0 (0.7–1.4)
Eating at school on the day of interview:			
Yes	85 (31.3)	220 (25.4)	1 (ref)
No	187 (68.8)	647 (74.6)	0.8 (0.6–1.1)
Eating out of home (frequency/week)			
None	17 (6.3)	164 (18.9)	1 (ref)
1–2 times/week	151 (55.5)	472 (54.4)	0.2 (0.2–0.3)**
2–5 times/week	66 (24.3)	189 (21.8)	1.2 (0.8–1.6)
>5 times/week	48 (17.7)	43 (4.9)	4.1 (2.6–6.5)**

* *P* < 0.05

** *P* < 0.001, (95% CI): 95% Confidence intervals, (ref) = reference group.

Dietary intake and food consumption frequency: The number of servings per day of different foods included in the questionnaire revealed that lean students consumed more servings of fruits; vegetables; and dairy products, including milk, while overweight and obese children consumed significantly higher servings of egg, potato (especially fried), carbonated soft drinks, sugary drinks, and sweet/candy per day [Table 3].

**Table 3:** Comparison of intake of selected foods items (servings per day) in children and its association with their BMI classification

Food items	Body mass index classification		*t*-Test, *P* value
		
	Obese and overweight (N = 272) No. (%)	Nonobese/nonoverweight (N = 867) No. (%)	
Green leafy vegetables	0.24 ± 0.36	0.39 ± 0.47	4.84, 0.002**
Other vegetables!	1.39 ± 1.05	1.98 ± 1.44	6.25, 0.001**
Fruits (include cocktail and mixed fruit)	0.61 ± 1.87	0.66 ± 2.51	0.30, 0.761
Fruits and vegetables	4.23 ± 2.77	5.30 ± 3.05	5.16, 0.001**
Milk and dairy products (include icecream)	1.91 ± 1.33	2.60 ± 1.56	2.77, 0.005**
Eggs	0.51 ± 0.65	0.42 ± 0.59	2.14, 0.032**
Juices (fruit and other drinks)	1.06 ± 1.96	1.04 ± 1.23	0.20, 0.841
Potatoes (fried, baked and cooked)	1.22 ± 0.87	0.98 ± 0.65	4.87, 0.001**
Carbonated soft drinks	1.43 ± 0.88	0.51 ± 0.78	16.45, 0.001**
Sugary drinks	2.16 ± 1.57	1.91 ± 1.36	2.55, 0.011**
Sweets and candy (include jelly, chocolate)	2.81 ± 2.78	2.11 ± 1.34	4.94, 0.001**
Meat products (any form including fast foods)	1.67 ± 1.35	1.70 ± 1.21	0.35, 0.728
Rice, pasta and pizza	0.64 ± 1.37	0.71 ± 1.18	0.82, 0.412
Packed foods (1)	0.34 ± 0.63	0.28 ± 0.41	1.83, 0.067
Legume (peas, beans and nuts)	0.82 ± 0.79	0.74 ± 0.71	1.58, 0.115
Other cereals*	0.63 ± 1.90	0.73 ± 1.81	0.79, 0.432
Bread (white and brown)	1.56 ± 1.19	1.41 ± 1.73	1.33, 0.182
Bakery products (donuts, cupcakes and biscuits)	1.54 ± 1.87	1.34 ± 1.68	1.67, 0.096

!Other vegetables include tomato, carrot, spinach, green peas and mixed vegetables

* Other cereals include breakfast cereals, oats, lentils and others, (1) Packed food include chips, popcorn, nuts, crackers, sweet rolls and others

** Statistically significant at 0.05 level.

Moreover, the frequency of eating selected food groups during the last week revealed that obese and overweight students frequently consumed meat and alternatives (48.9% vs. 39.8% in lean children), while less frequently consumed milk and milk products (12.9% vs. 56% in the lean children) (*P* < 0.001). On the other hand, lean children more frequently consumed fresh fruits (41.4% vs. 26.5%) and vegetables (39.4% vs. 36.8%); however, 34.5% and 36.5% of the included students stated a consumption of fresh fruits and vegetables for less than once per week [Table 4].

**Table 4:** Basic food group consumption as stated in frequency per week among the included primary schools students distributed according to their BMI classifications

Food group	Body mass index classification		Univariate analysis odds ratio and 95% confidence intervals
	
	Obese and overweight (N = 272) No. (%)	None (N = 867) No. (%)	
Meat and alternatives:			
≤Once/week	18 (6.6)	169 (19.5)	1 (ref)
2–4 times/week	121 (44.5)	353 (40.7)	1.2 (0.9–1.6)
5–6 times/week	133 (48.9)	345 (39.8)	1.5 (1.1–1.9)*
Milk, Cheese and other dairy products:			
≤ Once/week	69 (25.4)	143 (16.5)	1 (ref)
2– 4 times/week	168 (61.7)	248 (28.6)	4.0 (3.0–5.4)**
5– 6 times/week	35 (12.9)	485 (54.9)	0.1 (0.08–0.2)**
Fruits:			
≤Once/week	98 (36.0)	295 (34.0)	1 (ref)
2–4 times/week	102 (37.5)	213 (24.6)	1.8 (1.4–2.5)**
5–6 times/week	72 (26.5)	359 (41.4)	0.5 (0.4–0.7)**
Vegetables:			
≤Once/week	84 (30.9)	332 (38.3)	1 (ref)
2–4 times/week	88 (32.4)	193 (22.3)	1.7 (1.2–2.3)**
5–6 times/week	100 (36.7)	342 (39.4)	0.8 (0.7–1.1)
Bread and other bakery products:			
≤Once/week	12 (4.4)	52 (6.0)	1 (ref)
2–4 times/week	43 (15.8)	115 (13.3)	1.2 (0.8–1.8)
5–6 times/week	217 (79.8)	700 (80.7)	0.9 (0.7–1.3)
Rice and other cereals:			
≤Once/week	38 (14.0)	100 (11.5)	1 (ref)
2–4 times/week	34 (12.5)	156 (18.0)	0.7 (0.4–1.0)
5–6 times/week	200 (73.5)	611 (70.5)	1.2 (0.9–1.6)
Cooked vegetables:			
≤Once/week	99 (36.4)	349 (40.2)	1 (ref)
2–4 times/week	93 (34.2)	273 (31.5)	1.1 (0.8–1.5)
5–6 times/week	80 (29.4)	245 (28.3)	1.1 (0.8–1.4)

* *P* < 0.05

** *P* < 0.001.

The stated frequency of certain obesogenic food items per week among the different groups with regard to BMI showed that obese and overweight students were significantly reported to have higher frequency of soft drinks (OR = 3.4), although there is an apparent negative association between soft drink and obesity; after recategorization, overweight and obese subjects were reported to consume soft drinks at a higher frequency (60.3% daily or several per day vs. 30.9% among the lean subjects), sweets and candy (OR = 1.7, 49.3% vs. 35.8%), cakes/cookies/doughnut and similar foods (OR = 2.7, 49.6% vs. 27.1% in lean students) and potato chips/popcorn/other packed foods (OR = 5.9, 29.0% vs. 6.5% in lean students) [Table 5].

**Table 5:** The frequency of the selected obesogenic food consumption in the last week as stated by the presence of overweight and obesity in the primary school children

Food item frequency/week	Obesity and overweight		Univariate analysis odds ratio and (95% confidence intervals)
	
	Overweight and obese (N = 272) No. (%)	Nonoverweight/nonobese (N = 867) No. (%)	
Soft drinks (carbonated):			
1–2 times/week	53 (19.5)	324 (37.4)	1 (ref)
3–6 times/week	55 (20.2)	275 (31.7)	0.6 (0.4–0.8)*
Once or more/day	164 (60.3)	268 (30.9)	3.4 (2.5–4.6)*
Sweets/candy:			
1–2 times/week	77 (28.3)	328 (37.8)	1 (ref)
3–6 times/week	61 (22.4)	229 (26.4)	0.8 (0.6–1.1)
Once or more/day	134 (49.3)	310 (35.8)	1.7 (1.3–2.3)*
Cakes/cookies/doughnut/biscuits:			
1–2 times/week	71 (26.1)	324 (37.4)	1 (ref)
3–6 times/week	66 (24.3)	308 (35.5)	0.6 (0.4–0.8)*
Once or more/day	135 (49.6)	235 (27.1)	2.7 (1.9–3.5)*
Chewing gum:			
1–2 times/week	130 (47.8)	413 (47.6)	1 (ref)
3–6 times/week	117 (43.0)	343 (39.6)	1.1 (0.9–1.5)
Once or more/day	25 (9.2)	111 (12.8)	0.7 (0.4–1.1)
Chocolate:			
1–2 times/week	146 (53.6)	484 (55.8)	1 (ref)
3–6 times/week	103 (37.9)	345 (39.8)	0.9 (0.7–1.2)
Once or more/day	23 (8.4)	72 (8.3)	1.0 (0.6–1.7)
Potatoes chips/popcorn/packed foods:			
1–2 times/week	90 (33.1)	343 (39.6)	1 (ref)
3–6 times/week	103 (37.9)	467 (53.9)	0.5 (0.4–0.7)*
Once or more/day	79 (29.0)	57 (6.5)	5.9 (3.9–8.7)*
Pizza and similar food products:			
1–2 times/week	176 (64.7)	557 (64.3)	1 (ref)
3–6 times/week	86 (31.6)	293 (33.8)	1.2 (0.9–1.7)
Once or more/day	10 (3.7)	17 (1.9)	1.9 (0.8–4.5)

* *P* < 0.001.

### Sociodemographic and dietary predictors of obesity

Multivariate logistic regression model generated by the inclusion of socioeconomic variables and dietary habits, which are significant in the univariate analysis, by using the dependent variables overweight and obesity revealed that urban residence, older age of children, low maternal educational status, maternal occupational status, small family size and frequent consumption of food out of home are positively associated with the development of obesity and overweight; consuming breakfast at home was inversely associated with the development of outcome [Table 6]. The second logistic regression model generated by the inclusion of the frequency of consumption of food items significant at the univariate analysis showed that excessive consumption of carbonated soft drinks; sweet-candy; low consumption of vegetables, fruits and dairy products are possible predictors of the development of overweight and obesity among the included school children [Table 7].

**Table 6:** Multivariate logistic regression model for overweight and obesity and significantly independent variables (sociodemographic and dietary habits)

Covariates	β Coefficient	Multivariate analysis	
		
		Odds ratio (OR) and 95% confidence intervals (95% CI)	*P* value
Residence:			
Urban	0.811	1.85 (1.31–2.62)	0.011*
Rural	−0.342	1 (ref)	0.002*
Age groups:			
10–12 years	0.763	0.41 (0.31–0.54)	0.003*
12–14 years	0.448	2.1 (1.12–3.90)	0.020*
14 years	0.683	1 (ref)	0.014*
Maternal education:			
<Secondary	0.392	1.87 (1.23–2.49)	0.004*
Secondary or higher	−0.042	1 (ref)	0.018*
Working mother:			
Yes	0.258	1.85 (1.34–2.55)	0.033*
No	-	1 (ref)	-
Family size:			
≤6 per family	-	1.95 (1.15–3.31)	-
>6 per family	-	0.54 (0.33–0.89)	-
Taking breakfast at home:			
Yes	-	1 (ref)	-
No	-	1.76 (1.28–2.42)	-
Food away from home:			
>3 times/week	-	1 (ref)	-
≤3 times/week	-	-	-

* Statistically significant association, (ref): reference group, This model correctly predicts 68.6% of the cases. χ^2^ = 21.094, Constant = 3.159

**Table 7:** Logistic regression model of possible dietary intake revealed the significance after univariate analysis as potential predictors for obesity and overweight among the school children

Covariates	Coefficient β	Odds ratio (OR) and 95% confidence intervals (CI)	*P* value
Carbonated soft drinks:			
Once or more/day	0.159	(ref)	0.032*
Less	0.258	0.6 (0.50–0.8)	0.033*
Candy/sweets and baked foods:			
Once or more/day	−0.278	(ref)	0.018*
Less	−0.563	0.7 (0.6–0.9)	0.002*
Milk and dairy products:			
5–6 times/week	−0.449	(ref)	0.017*
<5 times/week	-	1.3 (1.1–1.6)	-
Fresh vegetables consumption			
5–6 times/week	-	1.8 (1.3–2.5)	-
<5 times/week	-	(ref)	-
Fresh fruits consumption			
5–6 times/week	-	-	-
<5 times/week	-	-	-

* Statistically significant at 0.05 level, (ref) = reference group, This model explained 70.8% of cases. χ^2^ = 18.732, Constant = 2.849

## Discussion

Economic development of Saudi Arabia during the last 3 decades has changed the nutritional and lifestyle habits;(21) food has become more affordable to a larger number of people with the substantial decrease in the price relative to income, and the concept of food has changed from a means of nourishment to a determinant of lifestyle and a source of pleasure, coupled with physical inactivity have likely contributed to the increase in the prevalence of overweight and obesity in the children.(16)

Our study revealed that the combined prevalence of obesity and overweight is 23.9% (obesity, 9.7% and overweight, 14.2%) among the included subjects.

In a household survey including children aged 1–18 years, the overall prevalence of overweight was 10.7% and obesity was 4.7% among the included males; the Eastern province had the highest prevalence compared to others in KSA,(15) while another school-based survey in the Kingdom revealed that the overall prevalence of overweight was 11.7% and obesity was 15.8% among the included male aged 6–18 years, and the highest prevalence of obesity was recorded in the capital Riyadh.(4)

Our results are higher than those reported in the household survey, while overweight in our study is in concordance with the previously mentioned school survey but lower with regard to the prevalence of obesity.

This difference could be explained on the basis of the different age groups included in these studies and/or the methods used for assessing overweight and obesity.

A study conducted in Italy reported a prevalence of obesity of 9.8% and overweight of 21.4% among school students aged 11–19 years,(21) while in Brazil, the prevalence of obesity and overweight among male school children aged 8–10 years were 7.4% and 17.3%, respectively.(22)

Our data as well as those of other studies(4,15–17) conducted in the Kingdom revealed a prevalence that approached or sometimes exceeded those reported in many developed countries. Wang,(23) reported a combined prevalence of overweight and obesity of 25.7% in the US, 11.5% in Russia and 5% in China in males within the age group of 10–18 years. This last notion implies the urgency for intervention to revert and reduce the epidemic of obesity and the possible health hazards with grave repercussions on adult populations and the health system.

Gillis and Bar(24) reported that obese children and adolescents consume significantly more servings of meat and alternatives, grain products, fast foods, sweetened soft drinks and potato chips, which contribute to increased deposition of calories, fat and sugar intake than that in nonobese children and adolescents.

Similar studies(25,26) have reported that overweight and obese children consumed more fats and less vegetables, fruits, legumes and dairy products.

Our results are in concordance with that of the previously mentioned studies since obese and overweight students in our study more frequently consumed meat and alternatives, soft drinks, sweets/candy and potato chips and less frequently consumed milk and dairy products those in the lean group; however, both groups consumed less fruits and vegetables, which was considerably less among the students in the obese group.

Moreover, our results revealed that in comparison to the recommended food consumption by the Healthy People Objectives 2010, that in the students in our study is extremely less;(25) these findings were also confirmed in the logistic regression model, which revealed that low consumption of fruits, vegetables, milk and dairy products are possible predictors of overweight and obesity among the students in our study.

A growing body of evidence suggests that increasing the dairy intake by approximately two servings per day could reduce the risk of overweight by up to 70%.(27)

In addition, calcium intake was associated with 21% reduced risk of development of insulin resistance among overweight younger adults and may reduce the risk of diabetes.(28) Higher calcium intake and more dairy servings per day were associated with reduced adiposity in children studied longitudinally.(27)

Several studies(13,14,22,24) indicated the association between less healthy eating habits and obesity in children. A school-based study in Brazil and other parts of the world have reported that missing or infrequent intake of breakfast and low frequency of milk consumption are positively associated with obesity and overweight as also noted in the primary students in our study.

Niklas *et al.*(13) argued that regular consumption of breakfast may control body weight due to the decrease in fat content in the diet because of the role it plays in minimizing the intake of high energy snacks. Children who eat breakfast consume a greater amount of grains, fruits and dairy products.

Our results are consistent with those of both the previous Brazilian study as well as Niklas, since obese and overweight students were significantly missing or infrequently taking breakfast compared to those in the nonobese group. In a study comparing the eating habits of obese to nonobese children, it was found that obese children consumed significantly more fast foods than the nonobese children. This has been shown to contribute a significant amount of extra calories and fat in the diets of obese adults.(24)

Our study reported a significant difference between obese and overweight children and the lean children with regard to the frequency of consumption of fast food.

In the logistic regression model, less healthy dietary habits were positively associated with obesity and overweight among the students in our study. These results are consistent with those reported in a similar study conducted on school children in younger age group in Brazil,(22) where less healthy eating habit was associated with a twofold risk of overweight and obesity.

A large number of studies on adults have examined the relationship between the socioeconomic status and obesity, but less studies have used the data to examine these relationships in children.(29,30) It was concluded that a strong inverse relationship exists between socioeconomic status and obesity among women in developed societies; however, this relationship is inconsistent for men and children.

In contrast, in developing countries, a strong relationship exists between socioeconomic status and obesity among men, women and children.(31) It is of concern, however, that since different definitions of obesity and indicators of socioeconomic status were used, the findings of different studies may not be comparable.(29)

In the current study, obesity and overweight were found to be associated with urban residence and low maternal educational status, which are consistent with the findings of other studies reporting a higher prevalence of childhood obesity among the low social class; however, reports on the association of obesity with low economic class are conflicting since our results revealed an association with maternal occupational status, which may be a proxy to higher economic status.

## Conclusion

The combined prevalence of overweight and obesity among the male children is increasing and is comparable to that found in the developed countries.

Less healthy dietary habits, poor selection of food and socioeconomic status may be associated with the problem of obesity and overweight among the school children assessed in Al-Hassa.

## Recommendations

Researchers involved in childhood obesity prevention may use the findings of our study to implement school-based food programs and nutritional health education messages with incorporation of skills for proper selection of food.

We emphasize the importance of breakfast, the hazards of eating out frequently and the importance of certain food items in the prevention of obesity.

Further studies are required involving females.

### Study limitations

We used the food frequency questionnaire that is subject to recall bias instead of detailed food diaries to calculate precisely the food consumption in terms of calories and other numeric measures.

The socioeconomic data collection through forms filled by parents may be amenable to errors of over and/r underreporting for which no quality control exists.
